# The Mechanism of Oxidative Stress in Cells Isolation, Identification, and Genome-Wide Sequence Analysis of Nitrite Amylolytic *Bacillus*

**DOI:** 10.1155/2022/9521900

**Published:** 2022-10-14

**Authors:** Jian Jiang

**Affiliations:** Department of Public Health, Jining Medical University, Jining, 272013 Shandong, China

## Abstract

To improve the quality of traditional fermented pickles and reduce the nitrite content in the production process of pickles, the target bacteria for efficient nitrite degradation were screened from traditional fermented pickles. Pickles (picked vegetables), a traditional dish favored by many Chinese, are mildly salted and lactic acid-fermented vegetables in China. However, the presence of nitrite in pickles is a bottleneck which limits further development of the pickle industry. More attention is drawn to the problem of the presence of nitrite in pickles. Having harmful effect in the acidic environment produced by gastric acid, nitrite is converted into carcinogenic nitrosamine. After screening several nitrite-degrading bacteria in the early stage, a Gram-positive round ended *Bacillus amyloliquefaciens* is named as *Bacillus amyloliquefaciens* JBA-CH9, which can degrade nitrite efficiently. *Bacillus amyloliquefaciens* is a common bacterium in the food fermentation industry. Then, the optimum conditions for nitrite degradation of the strain were explored according to the inoculation amount, temperature and salinity, and the whole genome of *Bacillus amyloliquefaciens* JBA-CH9 was sequenced. The results showed that the strain had the best degradation effect on nitrite under the conditions of inoculation amount of 9%, salinity of 5%, and 30°C, and the highest degradation rate of nitrite was 91.47%. The results of whole genome sequencing showed that the strain had a large number of functional genes related to amino acids, carbohydrates, and lipids and contained nitrite reductase genes related to nitrite metabolism. Therefore, *Bacillus amyloliquefaciens* JBA-CH9 is a functional strain that can degrade nitrite efficiently.

## 1. Introduction

Pickle is a unique fermented food in China with delicious taste, easy preservation, rich nutrition, and distinctive characteristics [1]. The production of pickles is a tedious process [2]. It is mainly the process of salting fresh vegetables to form low salt salted vegetable blank, and then putting the salted vegetable blank into a sauce jar with sauce, so that the salted vegetable blank absorbs the flavor substances in the sauce [3–6]. However, in the process of fresh vegetables becoming delicious pickles, the excessive nitrite produced by microorganisms still needs to be paid close attention [7]. Nitrite produced during fermentation adversely affects health due to formation of methemoglobin and conversion to carcinogenic nitrosamine. Excessive nitrite is a strong oxidizing agent. It oxidizes ferrous hemoglobin which transports oxygen in the blood to ferric hemoglobin. As a consequence, hemoglobin loses its oxygen transport capability leading to hypoxia. In the acidic environment produced by gastric acid, nitrite is converted into carcinogenic nitrosamine [8]. However, nitrite in moderation does not pose a major threat to human health, but acute large nitrite absorption can cause acute poisoning symptoms, including methemoglobin sickness. Nitrite can have teratogenic and carcinogenic consequences if consumed in large quantities or over an extended period of time [9–11]. The people hope to reduce the nitrite in pickles to a certain level and improve the quality of pickles. Therefore, the core goal of this study is to screen the active strains that can degrade nitrite efficiently from the traditional fermented pickles and use them in the production process of pickles.

Through numerous literature searches in the early stage, it was found that there had been many literatures on screening nitrite-degrading strains in pickles, and the screening of nitrite-degrading strains in traditional fermented pickles is rarely reported at this stage. The nitrite-degrading bacteria screened from pickles are mainly lactic acid bacteria with strong acid producing ability, and the degradation mechanism is relatively simple, most of them are acid degrading nitrite. The strains that have been found in the literature are mainly *Lactobacillus plantarum*, *Lactobacillus brevis*, *Lactobacillus casei rhamnosus,* and Screening, mutagenesis of nitrite and other strains [12–14]. At present, there are mainly two methods to degrade nitrite by strains. One is to produce acid by lactic acid bacteria, and then degrade nitrite by acid; the other is through the nitrite reductase producing strains, through the oxidation-reduction reaction to degrade nitrite. The present research focus is on finding strains with rapid growth and high nitrite-degrading activity for use in traditional fermented pickles [15–17]. Using the traditional strain separation approach, a highly active strain was chosen for this study, and the physiological, biochemical, and degrading activities of the chosen strain were assessed. The existing literature covers that whole genome sequencing is a mean to quickly understand the key functional genes (cell) related to a strain [18]. After the bacterial genome is sequenced and assembled from scratch, the genome circle map of the target strain can be formed, and the genome components, functional annotation, comparative genomics, and other bioinformatics analysis of the genes in the genome sequence can be carried out by using relevant software. It is to find out the key genes, cells, or enzymes related to the degradation of nitrite and preliminarily explore the mechanism of nitrite degradation. Therefore, there is no relevant report on the application of *Bacillus amyloliquefaciens* in the production of traditional pickles. Only in agriculture, *Bacillus amyloliquefaciens* can be used as an effective biological control strain [19–21]. In the process of sewage treatment and feed processing, *Bacillus amyloliquefaciens* also plays an important role [22–25]. To identify the key functional genes or cells related to nitrite degradation and provide a theoretical framework for the development of traditional fermented pickles, the bacteria isolated from traditional fermented pickles were separated, their nitrite degradation activity was assessed, and the strains with high degradation activity were sequenced and analyzed.

## 2. Methods

### 2.1. Medium

Samples of local pickles sold in Jining (provided by Jining Yutang sauce garden) contains Luria Bertani (LB) broth solid medium with 10 g tryptone, 20 g agar, 5 g yeast extract, 10 g sodium chloride, 1000 ml distilled water, and pH 7.0. LB liquid medium with 10 g tryptone, 5 g yeast extract, 10 g sodium chloride, 1000 ml distilled water, and pH 7.0; Distilled water; normal saline; Medical alcohol cotton ball; Iodine simple substance; 95% ethanol solution; Glycerol; Alcohol lamp; Soluble starch; LB broth; Agar.

### 2.2. Screening of Nitrite-Degrading Strains

Randomly cut 1 g from pickles, put it into a mortar, add corresponding normal saline according to the mass volume ratio of 1 : 10, fully grind it, stand for 15 min, and put it into an ultraclean workbench. Dilute pickle samples with normal saline according to the concentration gradient of 10^−1^ − 10^−3^ by the following process: prepare 6 Eppendorf tubes, number them, respectively, and prepare bacterial solutions of different concentrations in EP tubes. The strains with the best growth state and the largest single colony volume were selected from the plate and purified and screened repeatedly on LB solid medium. The strains to be tested were screened and inoculated into the liquid medium for culture. The bacteria were observed under the ordinary optical microscope, and the bacteria were stained with Gram before microscopic examination. According to the naphthalene ethylenediamine hydrochloride method in GB 5009.33-2016 national food safety standard, determination of nitrite in food and the screening strains' capacity to break down nitrite were assessed.

### 2.3. Physiological, Biochemical, and Molecular Biological Identification of Nitrite-Degrading *Bacillus Amyloliquefaciens* JBA-CH9

Inoculate the tested strain with hydrochloride degrading activity screened in 1.3.1 into LB agar medium after 2 generations of activation. After 24 hours of culture, observe the morphology of the strain. The physiological and biochemical characteristics of the strains to be tested were identified according to Berger's bacterial identification manual and detection and identification methods of *Bacillus subtilis* [26]. Based on the design and synthesis principle of 16S recombinant deoxyribonucleic acid (rDNA) identification primer, a general primer 27f:5′-agagtttgatcctggctcag-3′, 1492r:5′-cggttacctttgttacgact-3′ was designed according to the 16SrDNA gene sequence. The whole genome of the strain to be tested was extracted and isolated. 16S ribosomal ribonucleic acid (rRNA) bacteria were used for amplification through primers. The amplification system was a 25 ul polymerase chain reaction (PCR) system. The amplification reaction conditions were predenaturation at 94°C for 3 min, denaturation at 94°C for 30 s, annealing at 52°C for 1.5 min, extension at 72°C for 2 min for 30 s, 35 cycles, and total extension at 72°C for 10 min. The obtained sequences were compared by using the basic local alignment search tool (blast). The PCR products were sent to Sangong Bioengineering (Shanghai) Co., Ltd. for sequencing. The determined sequences were compared in the gene database by blast to identify species. At the same time, using Mega 7.0 software, the phylogenetic tree was constructed by adjacency method.

### 2.4. Response Surface Method Parameter Optimization

The effects of inoculation amount on (a) salinity, (b) temperature, and (c) nitrite degradation rate were investigated using response surface methodology (RSM). The RSM is a widely used mathematical and statistical method for modeling and analyzing a process in which response of interests is affected by various variables. In order to estimate the model coefficients, we conducted a three factor and three level central combination (BBD) experiment 17 times. The experimental sequence was random. The analysis of experimental design data and the calculation of predicted response were calculated by SPSS statistics 22.0. Subsequently, additional confirmatory experiments were conducted to verify the reliability of the statistical experiment design [27].

### 2.5. Sauce Fermentation

In order to prove its ability to degrade nitrite in the production of pickles and to evaluate its influence in the actual production of pickles, the *Bacillus amylolyticus* screened from pickles in Jining area was used. *Bacillus amyloliquefaciens* JBA-CH9 was inoculated into sterilized LB medium and cultured at 30°C for 24 hours to prepare fermentation seed solution; add 5% of the seed solution to the liquid LB medium to make the bacteria reach 10^7^–10^8^ colony forming unit (CFU)/ml, and then culture at 30°C for 24 hours without shaking to produce the secondary seed solution, which is the bacterial solution actually added to the pickle production process. Then, according to the fermentation process of the sauce, the cucumber embryo salted for 72 hours was washed, dried, cut into pieces, scalded, added with 5% secondary seed liquid and soybean sauce, and fermented in a sealed bottle at 37°C for 120 hours. During the whole production process, samples of pickled cucumber were collected regularly to detect nitrite concentration. The samples were not totally exposed to the air during the entire sauce fermentation process in order to maintain the stability of the fermentation flora. It was necessary to objectively assess the contribution of *Bacillus amyloliquefaciens* JBA-CH9 to the sauce fermentation process. The control group did not receive the *Bacillus amyloliquefaciens* JBA-CH9 inoculation and was instead fermented with regular sauce.

### 2.6. Whole Genome Sequencing of *Bacillus Amyloliquefaciens* JBA-CH9

Using the genome sequence (DNBseq) platform, genomic DNA was extracted and randomly interrupted. DNA segments of the required length were electrophoretically retrieved, prepared for gene clusters by splicing, and then sequenced on a computer. Then, the bacterial genome was de novo assembled after whole genome sequencing using the bacterial genome de novo sequencing method. The final assembly level was determined according to the needs of research and the characteristics of bacteria. According to the assembly level, it was divided into primary assembly, advanced assembly, and completion map assembly.

### 2.7. Genome-Wide Bioinformatics Analysis of *Bacillus Amyloliquefaciens* JBA-CH9

Using bioinformatics related software to analyze the genome components, after obtaining the sample assembly sequence, predict the functional elements in the sample genome including gene components, repeat sequences, and noncoding RNA. After the predicted genes, the genes need to be annotated by database comparison. Through sequence similarity, Gene Ontology (GO) and cluster of homologous groups of proteins (COG) are performed in the database.

## 3. Results

### 3.1. Isolation of *Bacillus Amyloliquefaciens*

Through the screening of bacterial colonies in the early stage, clear single colony strains with complete colony morphology can be seen in the solid nutrient plate. Through the observation of colony morphology, the colonies with good growth were examined by microscope. At the same time, the strains to be tested were stained with gram, and the strains to be tested were dyed blue purple under the ordinary optical microscope, which proved that the selected strains to be tested were all Gram-positive bacteria (Figure 1). Then, the strain with the largest single colony was selected as the strain to be tested for nitrite degradation, and the screened strains were numbered, respectively. Due to the degradation of nitrite, the strain needs to produce nitrite reductase before it can effectively degrade nitrite. Therefore, this requires the strain to have the key element of vigorous basic metabolism. To improve the success rate of screening nitrite-degrading strains in the next phase, the size of the formed colony can be used to screen the strain's growth and metabolism rate.

### 3.2. Identification of Nitrite-Degrading Strains

#### 3.2.1. Identification Experiment of Nitrite Degradation by Strains to Be Tested

Three strains AD1, AD7, AE5, BD3, BH2, CH6, CH9, DB8, and DC1 were selected for nitrite degradation evaluation. The ability of the three strains to degrade nitrite was tested by using the naphthalene ethylenediamine hydrochloride method in the national food safety standard—determination of nitrite and nitrate in food (GB 5009.33-2016). Three groups of parallel experiments were carried out for each strain. As time changed, the light absorption value of CH9 strain decreased significantly compared with the blank control. The average absorbance was only 0.158 indicating that CH9 strain had a strong ability to degrade nitrite. Compared with other strains, CH9 strain significantly reduced nitrite content. The results showed that the CH9 strain had the lowest level of nitrite in its culture medium, demonstrating that it had the greatest capacity to reduce nitrite. The following are the outcomes (Figure 2):

#### 3.2.2. Molecular Biological Identification of Nitrite-Degrading *Bacillus Amyloliquefaciens*

The 16S rDNA sequence and sequencing results of the strain CH9 to be tested were compared with blast similarity in the National Center for Biotechnology Information (NCBI). The strains of *Bacillus amyloliquefaciens* and *Bacillus subtilis* with high homology were selected, and the phylogenetic tree was constructed by the adjacency method. The results are shown in Figure 3. The construction of phylogenetic tree is a more comprehensive understanding of the genetic background of the screened *Bacillus amyloliquefaciens* JBA-CH9, and a more in-depth discussion on the mechanism of nitrite degradation by this strain in the later stage. It can be seen from Figure 3 that the strain CH9 to be tested is closely related to *Bacillus subtilis* 168.

### 3.3. Response Surface Methodology to Optimize Nitrite Degradation Rate

As shown in Table 1, the cross experiments of three factors and three levels were carried out, respectively. Using the three key factors of inoculum amount, salinity, and temperature, under the conditions of inoculum amount of 7%, salinity of 7% and temperature of 27.5°C, the maximum degradation rate of nitrite was 92.1% and 91.2%. However, when the inoculation amount was 2%, the salinity was 12% and the temperature was 27.5°C, and the degradation rate of nitrite was only 50.1%. It showed that the inoculum amount and salinity had a significant effect on the degradation rate of nitrite by CH9 at the same temperature. The response surface curve 3D (Figure 4) shows the comprehensive effect of different factors on the response (nitrite degradation rate). The experimental data conforms to the equation. The optimal operating parameters determined according to the equation are (a) inoculation amount 9.1%, (b) salinity 5.41%, (c) temperature 30.19°C, and (d) nitrite degradation rate 91.47%.

### 3.4. Dynamic Change of Nitrite Concentration during Sauce Fermentation

The effect of inoculation of *Bacillus amyloliquefaciens* JBA-CH9 on nitrite concentration of fermented cucumber embryo is shown in Figure 5. After 24 h and 48 h of fermentation, the nitrite content in Cucumber embryos without JBA-3 inoculation was 18.35 mg/kg and 51.26 mg/kg, respectively. The nitrite content in Cucumber embryos inoculated with *Bacillus amyloliquefaciens* JBA-CH9 decreased to 1.75 mg/kg and 0.89 mg/kg, respectively. After 72 hours of fermentation, the nitrite concentration in Cucumber embryo further decreased to 0.76 mg/kg and stabilized at this level. The nitrite concentration in Cucumber embryos inoculated with *Bacillus amyloliquefaciens* JBA-CH9 was significantly lower than that of noninoculated CH9 (*p* < 0.01). The nitrite concentration in fermented pickles not inoculated with *Bacillus amyloliquefaciens* JBA-CH9 showed a curve of first increasing and then decreasing and reached the maximum nitrite concentration of 51.26 mg/kg after 48 hours of fermentation. It can be seen that *Bacillus amyloliquefaciens* JBA-CH9 can significantly inhibit the abnormal accumulation of nitrite during the fermentation of pickles. With the continuous accumulation of nitrite in the fermentation process of pickles, the nitrite concentration in pickles decreased significantly when *Bacillus amyloliquefaciens* JBA-CH9 was added. In the control group, the high concentration of nitrite was maintained for a long time without the addition of *Bacillus amyloliquefaciens* JBA-CH9.

### 3.5. Sequencing Results of the Whole Genome of *Bacillus Amyloliquefaciens* JBA-CH9

The genomic DNA of *Bacillus amyloliquefaciens* JBA-CH9 was extracted through the DNBseq platform, and the bacterial genome was de novo assembled after the whole genome was sequenced through the bacterial genome de novo sequencing method. Eventually, the entire CH9 genome sequence was retrieved, and the Circos software was used to create a genome circle map with the entire genome sequence (as shown in Figure 6). *Bacillus amyloliquefaciens* JBA-CH9 has a genome that is 4387814 base pairs long, 4833 genes, a GC content of 45.97%, and a total gene length of 3850938 base pairs.

### 3.6. Analysis of Genome Components of *Bacillus amyloliquefaciens* JBA-CH9

By analyzing the distribution of each functional element, we can have a more in-depth study on *Bacillus amyloliquefaciens* JBA-CH9. The composition of noncoding RNA can play a role of regulatory factors in bacterial metabolism and environmental adaptation. Through the analysis in Table 2, we found that the copy number of tRNA was 87, that of 5SRNA, 16SRNA, and 23SRNA were 9, and that of sRNA was 41.

### 3.7. Annotation of Functional Genes in the Genome of *Bacillus Amyloliquefaciens* JBA-CH9

A protein sequence in the screened strains can be annotated into a protein homologous cluster by the comparison of sequencing genes; each COG cluster is made up of lineal homologous sequences, and the function of the gene can then be determined. Through COG analysis, we found that there were 319 genes related to amino acid transport and metabolism, 259 genes related to carbohydrate transport and metabolism, and 166 genes related to energy metabolism (Figure 7). Through functional gene annotation, we found that JBA-3 strain has a large number of functional genes related to amino acids, carbohydrates, and lipids, indicating that the strain has high activity in the processing and transport of nutrients.

The genes of *Bacillus amyloliquefaciens* JBA-CH9 can be divided into three categories based on their similarities to those in the go database: cytological component, molecular functional component, and biological pathway. Through the comparative analysis of go database, we found that there were 1427 genes related to catalytic activity, including the key gene related to nitrite metabolism - nitrite reductase gene, which was analyzed in-depth. This gene was a nitrite reductase ferredoxin like domain. There are 226 genes related to transport activity and 123 genes related to transcriptional regulation activity (Figure 8). Through the comparison of go database, we found that *Bacillus amyloliquefaciens* JBA-CH9 has genes related to nitrogen utilization and metabolism. The most important discovery is that *Bacillus amyloliquefaciens* JBA-CH9 contains nitrite reductase gene, which is the key gene for nitrite degradation. Through further analysis, the strain maintains high activity in the process of nutrient transport and transcriptional regulation.

## 4. Discussion

In this experiment, a strain of *Bacillus amyloliquefaciens* JBA-CH9, which can degrade nitrite efficiently, was successfully screened from the traditional fermented pickles, and the morphology of the screened strain was observed. Through the evaluation of nitrite degradation activity, the most active strain was screened. Then, the response surface methodology was used to optimize the optimal culture conditions for the strain to degrade nitrite, and the degradation rate of nitrite was improved. Finally, the whole genome of the strain was sequenced by DNBseq platform, and the genomic components and functional genes of the screened *Bacillus amyloliquefaciens* JBA-CH9 were analyzed.

The strain has the ability to degrade nitrite efficiently, and the degradation rate of nitrite can reach 91.47%. According to the evolutionary history of the strains, *Bacillus amyloliquefaciens* and *Bacillus subtilis* have a high genetic relationship. In recent years, *Bacillus amyloliquefaciens* has been isolated from *Bacillus subtilis*. *Bacillus amyloliquefaciens* has a strong ability to decompose starch and can produce the ability to inhibit the secondary metabolites of fungi and bacteria. Therefore, *Bacillus amyloliquefaciens* is a food grade strain with good industrial application prospects.

Although *Bacillus subtilis* is not the predominant bacterium during the traditional pickle fermentation process, the strains selected this time are capable of degrading nitrite effectively. Therefore, by enhancing *Bacillus amyloliquefaciens* JBA-CH9, we may change the traditional production process in the fermentation of sauce and regulate the nitrite produced in the production of pickles. In the later stage, by improving the existing pickle production process, nitrite-degrading bacteria were added during the fermentation period to control the accumulation of nitrite in pickles to the greatest extent. Finally, it makes pickles safer to eat, richer in taste and flavor, and improves the economic benefits of pickles.

## 5. Conclusion

Pickle is a traditionally popular food in China and exhibits health-promoting effects. However, there is a serious concern that nitrite produced during fermentation adversely affects health due to formation of methemoglobin and conversion to carcinogenic nitrosamine. The core goal of this study is therefore to screen the active strains that can degrade nitrite efficiently from the traditional fermented pickles and use them in the production process of pickles. A strain of *Bacillus amyloliquefaciens* JBA-CH9, which can degrade nitrite efficiently, was successfully screened from the traditional fermented pickles by observing the morphology of the screened strain. The strain has the ability to degrade nitrite efficiently, and the degradation rate of nitrite can reach 91.47%. Under the detailed mechanism given in ‘discussion section', the whole genome of the strain was sequenced by DNBseq platform, and the genomic components and functional genes of the screened *Bacillus amyloliquefaciens* JBA-CH9 were analyzed to achieve desired results.

## Figures and Tables

**Figure 1:** Gram staining and microscopic examination of *Bacillus amyloliquefaciens.*

**Figure 2:** Evaluation of nitrite degradation ability of screened strains.

**Figure 3:** Phylogenetic tree of *Bacillus amyloliquefaciens.*

**Figure 4:** 3D diagram of response surface curve.

**Figure 5:** Changes of nitrite concentration during soy sauce fermentation.

**Figure 6:** JBA-CH9 genome map.

**Figure 7:** Annotation distribution map of COG functional genes.

**Figure 8:** Annotation distribution map of GO functional genes.

**Table 1:** Factor level table.

Run	Inoculation quantity	Salinity	Temperature	Nitrite degradation rate
	%	%	°C	%
1	7	7	27.5	92.1
2	7	7	27.5	91.2
3	2	2	27.5	75.3
4	12	7	40	65.2
5	12	12	27.5	80.8
6	7	12	15	62.6
7	12	2	27.5	90.2
8	7	7	27.5	89.9
9	7	2	15	75.7
10	7	7	27.5	85.4
11	7	2	40	59.9
12	2	7	40	55.4
13	2	7	15	62.3
14	7	12	40	71.5
15	7	7	27.5	86.2
16	2	12	27.5	50.1
17	12	7	15	75.7

**Table 2:** Analysis of noncoding RNA components of JBA-CH9 genome.

Sample name (#)	Type (#)	Copy number (#)	Average length (bp)	Total length (#)	% in genome
JBA-3	tRNA	87	77.13	6,711	0.1529
	5s_rRNA (Denovo)	9	115	1035	0.0235
	16s_rRNA (Denovo)	9	1,538	13842	0.3154
	23s_rRNA (Denovo)	9	2,928	26352	0.6005
	sRNA	41	91.75	3,762	0.0857

## Data Availability

The data underlying the results presented in the study are available within the manuscript.
